# Effects of Variable Composite Attachment Shapes in Controlling Upper Molar Distalization with Aligners: A Nonlinear Finite Element Study

**DOI:** 10.1155/2021/5557483

**Published:** 2021-08-20

**Authors:** Cengiz Ayidağa, Beste Kamiloğlu

**Affiliations:** Department of Orthodontics, Faculty of Dentistry, Near East University, Near East Boulevard, Nicosia-Northern Cyprus, Mersin 10, Turkey

## Abstract

The objective of the present study is to describe the stress and displacement patterns created by clear aligners and composite attachments bonded with the acid-etch technique on the labial surface of the maxillary first upper molar during its distalization. Maxillary molar distalization is a clinical orthodontics procedure used to move the first maxillary molar distally. The procedure is useful in patients with some Class II malocclusion allowing the first molar to move into a Class I relationship and the correction of associated malocclusion features. Three finite element models were designed to simulate the alveolar bone, molar tooth, periodontal ligament, aligner, and composite attachments. The first model had no composite attachment, the second model had a vertical rectangular attachment, and the third model had a newly designed attachment. A loading method was developed that mimicked the aligner's molar distal movement. PDL was set as a viscoelastic material with a nonlinear mechanical response. von Mises and maximum principal stresses and tooth displacement patterns were analyzed using dedicated software. All the configurations showed some form of clockwise rotation in addition to the distal movement. The crown portion of the tooth showed maximum displacement in all three models; however, in the absence of attachment, the root apex moved in the opposite direction which was compatible with uncontrolled tipping movement. Simulations with attachments exhibited the best performance regarding the movement patterns. The third group, with the newly designed attachment, exhibited the best performance concerning stress distribution (principal stress and von Mises stresses) and higher stresses in the periodontal ligament and tooth. Incorporating a vertical rectangular attachment in a clear aligner resulted in the reduction of mesiodistal tipping tendency during molar distalization. The third model was the most efficient considering both displacement pattern and stress distribution. The level of stress generated by the third model needs to be further investigated in future studies.

## 1. Introduction

Class II malocclusion represent a large and heterogeneous group of malocclusions. Based on sagittal (horizontal) dental and skeletal variables, Moyer et al. identified 6 Class II subgroups [1]. Type A is characterized by the absence of skeletal discrepancy and maxillary dentoalveolar protrusion, thus requiring distalization of the maxillary dentition to establish a Class I molar/canine relationship and a normal overjet [2]. Molar distalization is a term used to describe the distal movement of the molars resulting in lengthening of the dental arch, in order to gain space in the maxillary arch. Distal movement should ideally be translatory (bodily tooth movement) where the crown and root move simultaneously as opposed to tipping where only the crowns move while the root tip is stationary [3]. In order to achieve bodily movement, the force should be applied at the center of resistance of the tooth. It has been experimentally determined that the center of resistance of the upper first molar passes slightly occlusal to the furcation of the roots [4].

Different appliances have been used for upper molar distalization, the most common being the headgear that uses extraoral traction that has several advantages but requires significant patient cooperation to be effective [5]. Alternative appliances have been used to move molars distally with reduced compliance requirements. The majority of these appliances, with very few exceptions, are not able to produce bodily molar movement since the line of force hardly passes through the center of resistance of the maxillary molars showing significant molar tipping [5]. With fixed orthodontic appliances, the force system that results in orthodontic tooth movement is produced by the interactions of metal wires and brackets attached to the tooth. Although with fixed appliances the forces are usually applied to attachments on the buccal surfaces of teeth, body movement is achieved by applying a force and a counter movement to prevent tipping [3].

It has been suggested that the force system generated by clear aligners, the most recently introduced class of orthodontic appliances, can mainly tip or intrude teeth but pure translation is not possible, at least theoretically [6]. However, Simon et al. investigated the force system generated by aligners in an experimental study and found that aligners can deliver the necessary force system to obtain bodily tooth movement [7]. Furthermore, molar distalization was the most predicable movement based on the results of a systematic review that assessed the predictability of orthodontic movements of teeth with aligners [8]. Clear aligners have evolved developing auxiliary elements such as composite attachments to control the quality of tooth movement [3]. It has been suggested that composite attachments can also produce counter moment to achieve bodily movement [3]. Few studies have been published that assessed the clinical and biomechanical performance of aligners and composite attachments during maxillary molar distalization.

In a retrospective clinical study, molar distalization presented the highest accuracy, approximately 87%, compared to incisor torquing and premolar derotation [9]. The correct staging (movement per aligner), but not the use of attachments, significantly impacted clinical efficiency [9]. Previously published studies, mainly case reports, have reported the possibility of achieving correction of Class II malocclusions by upper molar distalization with aligners even without attachments [10, 11]. Two studies, a case-control and a retrospective cohort, found that the use of composite attachments influenced the force level and tooth movement and was important in increasing the efficacy of molar distalization [12, 13]. The use of vertical attachments resulted in distal movement of the upper molars without significant tipping of the distalized molars [13]. In these clinical studies, the bodily moment was assessed based on the superposition of pretreatment and posttreatment cephalograms, a method prone to measurement errors.

Finite element methods have been employed to assess the biomechanics of bodily tooth moment with aligners and the role of composite attachment in displacement patterns [14–17]. Gomez et al. suggested that bodily movement of the tooth is more likely to occur in the presence of attachments [14]. Attachments produced a counter moment that counteracts the tipping tendency when the aligner segment is displaced distally without attachments [14]. Comba et al. investigated the effect of composite attachments combined with Class II elastics on upper canine distalization. The use of vertical rectangular attachments produced tipping movement while the use of optimized attachments produced bodily movements [15]. Yokoi et al. evaluated the effect of composite attachments on the bodily movement of central incisors during diastema closure demonstrating that the attachments were effective for achieving bodily movements [16]. The only FE analysis that assessed the molar distalization concluded that despite the force level and the amount of tooth displacement being influenced by attachments use, these are not sufficient alone to achieve distalization of the upper molars [17].

The present study aims to describe, using a FE model, the stress and displacement patterns generated by aligners and auxiliaries' composite attachments during upper molar distalization and the effect of a new composite attachments' shape and orientation in controlling this movement.

## 2. Materials and Methods

This research was conducted at the Department of Orthodontics, Faculty of Dentistry, Near East University (Northern Cyprus).

Three FE models were developed to simulate the alveolar bone, teeth, periodontal ligament (PDL) aligners, and attachment (Figure 1). The first models were with no composite attachment, and the second was with a vertical rectangular attachment positioned on the buccal surface of the maxillary 1^st^ molar. The third model was with the guideline attachment positioned on the buccal surface of the first maxillary molar.

Teeth, comprising the crown and the root, were designed based on ideal anatomy and position, with a mesiodistal angulation of 5.73 degrees, and labiolingual inclination of −11.3 degrees [18]. PDL was modelled by adding 0.2 mm of the tooth root. The thickness variability of PDL was not considered since it was modelled as a uniform layer [14]. Images obtained from cone-beam computed tomography (CBCT) data were used to reconstruct the alveolar bone. The upper jawbone of an adult edentulous patient was scanned using CBCT (ILUMA, Orthocad, CBCT, 3M Imtec, Oklahoma, USA). The patient was not involved in the experiment directly since the exam was prescribed retrospectively outside of the study's context. Permission was requested and the medical images were properly deidentified, before use. CBCT data were processed using 3D-Doctor software (Able Software Corp., Lexington, Massachusetts, USA). Dimensional and topographic adjustments of the jaw model were made in VRMesh software (Virtual Grid Inc, Bellevue City, WA, USA). Root shapes were excluded from the alveolar bone model and replaced by the designed model; in this way, each tooth can be independently manipulated. CAD procedures were used to design the aligner and attachment shape. Aligner thickness was set at 0.3 mm [14]. Aligner shape was developed by matting dental crown surfaces. Attachments were designed as vertical rectangular attachments with 2.75 mm height, 1.75 mm width, and 1 mm thickness and the guideline attachment with 1.8 mm height, 4 mm width, and 1 mm thickness (Figures 2 and 3). The guideline buccal attachment was designed as a half-round at a cross section. The orientation of the attachment presented 5 degrees of inclination regarding the horizontal plane with the distal extreme located occlusally. We hypnotized that this design of the attachment would introduce a counterclockwise moment produced by forces on the active surfaces of the attachment that will add to the moment generated by the tooth-aligner system. After CAD design with VRMesh Studio, all components were imported for FE analysis in the ALGOR FEMPRO (ALGOR, Inc. 150 Beta Drive Pittsburgh, PA 15238-2932 USA) software.

Model detail verification and convergence tests are possible with surface modelling tools (Surface-First Approach) for parametric modelling. However, we have used mesh surface modelling (Mesh-First Approach) to get highly detailed and realistic organic 3D models that cannot be achieved by parametric surface modelling. The software that we have used can import the mesh models (.stl files) and perform solid modelling and analysis. This method has the advantage of working on highly realistic 3D models compromising the ability to find the convergence point. However, since our models are highly detailed and the number of mesh nodes is far beyond any possible convergence point, we assume that we overcame that disadvantage of the Mesh-First Approach method.

The physical properties of each structure, apart from the PDL, were described by using a linear elastic model. The alveolar bone and teeth were modelled as an isotropic nonhomogenous material with a linear elastic mechanical response. It is important to select individual material properties that align with the study goals to obtain accurate results in the region of interest [19]. In the present study, a nonlinear, time-dependent viscoelastic model of the PDL was adopted, as proposed by Qian et al. [20]. It has been suggested that due to the higher stiffness of the tooth and bone compared to the PDL tissues, the assumption of linearity does not affect the final results [21]. Cataneo et al. suggested that the nonlinear response of the PDL may not need to be addressed while performing an analysis of the first phase of the orthodontic reaction as in the present study [22]; however, a more complex model guarantees more realistic results [23]. The behaviour of the aligner was also considered linear elastic [24]. The aligner thickness was 0.30 mm, and the material was also set as isotropic and homogenous. The attachments are made of composite material. The material properties were set as isotropic and homogenous, based on values reported in previous studies [14].  Table 1 summarizes the material properties assigned to each structure.

With regard to the coordinate system adopted in the present study; *y*-axis represents the sagittal plane with the positive direction being toward the mesial surface of the tooth and *z*-axis represents the vertical dimension with the positive direction toward the apical part.

Bonded contacts, corresponding to a perfect rigid union (no degrees of freedom) between contact surfaces, were used to join the spongious and cortical bone, cortical bone-PDL, and tooth-attachment interface. Tooth and PDL were relatively constrained by bonded contact, which only allows small sliding movements between joined nodes. Also, the bone extremities were fixed in every direction (on the mesial, distal, buccal, and palatal boundary surfaces) (Figure 4). The interface between the aligner and the tooth was modelled by using a friction model [10]. The coefficient of friction between tooth crown and aligners was set at 0.2 as reported in previous studies [11].

The aligner was restricted along the *y* (−) axis, *z* (−/+) axis, and *x* (−/+) axis in the study to avoid any dependencies on force direction and calculations for anchorage and to prevent any potential differentiation in the future studies. Movement can be described as 0.15 mm displacement along the *y* (+) axis. The load was introduced by moving the tooth distally by 0.15 mm. To generate a loading condition, an initial penetration between the target tooth and the aligner is necessary. This loading condition described here is the opposite of what occurs in a clinical setting, where the aligner is thermoformed in the printed model with the maxillary first molar already distalized and the force system that results in tooth movement is produced by this mismatch.

Outcome analysis in this study included the following:

1. von Mises stress
2. Tension-compression pattern at the PDL
3. Displacement pattern

## 3. Results

Displacement magnitude, distribution of von Mises stresses on the tooth, and maximum principal stress on the PDL, after application of a 0.15 mm displacement at the level of the first upper molar, are presented in Figures 5–7.

In the present study, negative sign for the maximum principal stress analysis indicates compressive stresses and positive sign, tensile stresses. In the first group, without attachment, the tensile stresses were higher in the cervical half of the mesial root surface (6.5 MPa) and cervical third of the distal root surface. Highest compressive stress (−0.43 MPa) was concentrated at the distobuccal aspect of the distal root. Compressive stresses were observed in both the mesial and distal aspect of the apical part of the palatal root, supposedly due to the rotation of the tooth (Figure 5). When a vertical attachment was added to the tooth crown, similarly highest tensile stresses were observed in the cervical-mesial aspect of the distal root (6.3 MPa). Tensile stresses were observed in the distal aspect of both the mesial and distal root. Tensile forces were less uniformly distributed compared to the first group. Furthermore, small compressive forces were developed on the distal aspect of both buccal roots (Figure 5(b)). Compressive stresses were uniform at the distal aspect of the three roots for the third group with guideline attachment. Maximum tensile stress was recorded in the cervical part of the mesiobuccal root (6.8 MPa). Highest compressive stresses were recorded in the mesial part of both buccal roots. More even stress distribution was observed in the distal side in the third group (Figure 5(c)).

von Mises stresses at the tooth level predicted by the FE models of the first maxillary molar for the three groups and the displacement magnitude are presented in Figures 6(a)–6(c). von Mises stresses were significantly higher at the apex of the three roots in the nonattachment group compared to the vertical attachment group (Figures 6(a) and 6(b)). High von Mises stresses were observed at the furcation level for the first two groups. For the third group, higher von Mises stresses were predicted by the third simulation at the apex level (Figure 6(c)).

The maximum displacement was observed at the crown level for all the groups (Figure 7). The movement of the maxillary molar was magnified 10 times with respect to the actual displacement. In the no-attachment group, the apical part of the palatal root was displaced mesially suggesting uncontrolled tipping movement (Figure 7(a)).

The standard aligner led to the lowest desired translation on the *y*-axis, and to the highest undesired movement, the palatal root was displaced mesially (−0.002 mm) suggesting uncontrolled tipping movement (Figure 7(a)). The maximum tooth displacement along the *y*-axis was obtained with the guideline buccal attachment, which showed 0.13 mm of translation at the coronal level, 0.1 mm at the furcation level, and between 0.07 and 0.08 mm at the root apex of all three roots. Displacement obtained with the vertical rectangular buccal attachments showed 0.13 mm of translation at the coronal level, 0.09 mm at the furcation level, and 0.05 mm at the level of each root apex. The lowest tooth displacement was obtained with the standard aligner configuration i.e., without attachments, showing 0.12–0.13 mm of translation at the coronal level, 0.076 mm at the furcation level, and between 0.01 mm at the level of each root apex (Figures 7(b) and 7(c)). In the guideline attachment group, the degree of distal root movement increased with respect to the vertical attachment group which was more evident for the distal root; still, the difference in the level of displacement between the crown and apical portion of the root was not uniform, indicating a certain degree of controlled tipping (Figures 7(b) and 7(c)).

This result can be related to the different angles between the attachment active surface and the tooth. Further studies should also investigate the effect of the attachment positioning criteria on the tooth movement, focusing on the amount of active surface of the attachment.

## 4. Discussion

Despite the increasing popularity of clear aligners, a discrepancy is often observed between the actual outcomes and the planned orthodontic movements in virtual setup [25, 26]. This may be due to an inadequate force system generated by the aligner but also aligner deformation in the mesiobuccal direction upon insertion, which may be accounted by the loss of programmed tooth movement [17].

Aligners alone are not suitable for obtaining bodily movement as demonstrated for the palatal and labial translation of the upper incisor tooth [27]. Attachments represent necessary auxiliaries used to aid in obtaining complex orthodontic movements [28]. A possible mechanism of action is through a local increase of the mismatch in specific areas, accurate control of load intensity and direction etc. Gomez et al. hypnotized that the attachments on the buccal aspect of the tooth helped counteract the inclination tendency by producing a countermoment that favours bodily translation, while in the absence of an attachment, a clockwise moment is produced which results in distal tipping of the tooth [14].

The effectiveness of attachments in producing bodily tooth translation has been demonstrated in previous FE model studies [14–17, 24]. Optimized attachment can control the tipping of the canines and central incisors during translation movement with aligners. Comba et al. found that not only the optimized attachments were effective in producing bodily movement of canine but also the vertical attachment produced buccal root displacement which may result in periodontal support damage [15]. Furthermore, the attachment geometry/orientation, horizontal vs vertical configuration, influenced the force system at the tooth level [24]. Vertical rectangular attachments are routinely used in clinical practice to support complex tooth movements; however, little evidence has been published to support their effectiveness during maxillar molar distalization.

The results of the present analysis suggest that uncontrolled tipping occurred when aligners moved the tooth in the absence of attachment. The addition of a vertical rectangular attachment resulted in a distal movement of the apexes of the roots. Still, the maximum displacement was observed at the crown level for both groups with an attachment, suggesting some degree of mesiodistal tipping. Principal stresses were determined at the periodontal ligament. In the third group, with guideline attachment, the stress was distributed more uniformly through the length of the root of the tooth, showing a pattern seen during maxillary first molar translation [29]. In all analyzed configurations, some degree of tipping occurred during molar distalization. Pure bodily translation with full control of tipping cannot be possibly achieved with any orthodontic appliance, but what we should be aiming is to control and eventually correct the tipping effect using additional mechanical procedures [30]. Comparison between groups concerning stress values may be obtained from the interpretation of the stress patterns rather than peak stress values considering the nonlinear assumption of PDL proprieties. The principal idea behind the production of the attachment in the third group was the existence of 2 active surfaces for obtaining moment. Moreover, a cylindrical horizontal body was considered to increase the connection between the aligner and the tooth.

Compared to other experimental models, FE analysis considers PDL so the assignment of the tissue properties can influence the stress values and distribution patterns as demonstrated by previous reports. In general, the linear model can underestimate PDL principal stresses and von Mises stresses at the root and overestimates them at the mid-root location [31]. We did include a comparative analysis concerning stress magnitude since the stresses in nonlinear models are higher than those calculated by linear models [31], and to our knowledge, this is the first study that considered the molar distal movement using a nonlinear FE analysis.

The current simulation is limited to the stress and movement analysis in the sagittal plane. Future simulations should consider other planes. Clinical experience suggests that the aligners can effectively control mandibular divergence during molar distalization [32]. This is particularly relevant in controlling vertical dimension when treating Class II patients with hyperdivergent growth pattern and anterior open bite.

Furthermore, in the present FE model, the analysis is limited to a single tooth. The results assume that the first molar has an ideal angulation and inclination and normal marginal bone levels. Most of the FE studies on clear aligners are limited to a single tooth, or at times, a segment of the dental arch and only a few have established complete dental arch models. Previous research has shown that the extension of the segment included in the analysis influences, although to a small degree, the biomechanical response of the PDL [33]. This is most likely caused by a difference in boundary condition settings [33]. However, in our analysis, a large area was modelled, and the boundary conditions were applied farther from the tooth that needs to be moved. Considering the effect of molar distalization on the entire arch will provide invaluable information on the responses of various units to the application of orthodontic forces. Rossini et al. studied the effect of different attachment configurations during upper molar distalization with aligners. Maximum displacement was observed for the lateral incisors in the model without attachments. It can be assumed that the attachments placed from the molar to canine would act as anchorage counteracting the undesired buccal flaring of the incisors during molar distalization [17]. In addition, Ravera et al. found that distal movement of the first molar in the absence of a vertical rectangular attachment on the second maxillary molar resulted in significant tipping of the first molar [13].

The results of this simulation are limited to the analysis of stress and displacement patterns during initial tooth movement. However, tooth movement is a dynamic long-term process accompanied by an alteration of the force system and mechanical response of the tissues. Tooth movement and force generated by the aligners were maximal at the beginning of the process and quickly decrease [34]. The change in force during tooth movement may be exponential as reflected by the changes in the highest PDL stress and maximum displacement values. This may have several implications. For example, Yokoi et al. found different displacement patterns for static and dynamic tooth movement simulation of central incisors during diastema closure. Incisors tipped and rotated during initial force application and bodily movement was observed after loading was applied for a long time after a sufficiently long [16].

Future FE models might take into consideration the effect on the entire arch and the dynamic nature of tooth movement, and experimental studies that verify the reliability of the present FE model should be carried out in the future.

## 5. Conclusions

This FE analysis was developed to assess the effect of different attachment configurations on the efficacy of bodily movement of the upper maxillary molar. The results show that configuration without an attachment and with a vertical rectangular attachment produced inclination of the molar in the mesiodistal direction while the guideline attachment produced stress and displacement pattern that most resembles bodily movement.

## Figures and Tables

**Figure 1:** Finite element model of the tooth and supporting structures.

**Figure 2:** Dimensions of the composite attachments.

**Figure 3:** Geometrical configurations of composite attachments in correspondence of the labial tooth crown surface. (a) Vertical rectangular attachment; (b) guideline attachment.

**Figure 4:** Boundary conditions.

**Figure 5:** Maximum principal stress in the first maxillary molar periodontal ligament during 0.15 mm distalization for the three groups: (a) without attachment, (b) with rectangular vertical attachment, and (c) with guideline attachment.

**Figure 6:** von Mises stresses distribution in the root and crown of the first maxillary molar for the three groups: (a) without attachment, (b) with rectangular vertical attachment, and (c) with guideline attachment.

**Figure 7:** Displacement patterns of the root and crown of the first maxillary molar for the three groups: (a) without attachment, (b) with rectangular vertical attachment, and (c) with guideline attachment.

**Table 1:** Mechanical properties of the involved structures.

	Young's modulus (MPa)	Poisson's ratio	References
Cortical bone	13.7 × 10^3^	0.30	Barone et al. [23]
Spongious bone	1.37 × 10^3^	0.30	Barone et al. [23]
Composite attachment	12.5 × 10^3^	0.36	Gomez et al. [14]
Plastic aligner	528	0.36	Gomez et al. [14]
Enamel	4.1 × 10^4^	0.30	Gomez et al. [14]
PDL (nonlinear elastic)^*∗*^		0.45	Qian et al. [20]

PDL, periodontal ligament. ^*∗*^Nonlinear mechanical properties for PDL were based on experimental data.

## Data Availability

The data underlying the findings of the study are available from the corresponding author upon request.
